The article "STK35 Gene Therapy Attenuates Endothelial Dysfunction and Improves Cardiac Function in Diabetes" was retracted in 2023. Reasons: duplicated images; unreliable data; unreliable results or conclusions.

# STK35 Gene Therapy Attenuates Endothelial Dysfunction and Improves Cardiac Function in Diabetes

**DOI:** 10.3389/fcvm.2021.798091

**Published:** 2022-01-13

**Authors:** Darukeshwara Joladarashi, Yanan Zhu, Matthew Willman, Kevin Nash, Maria Cimini, Rajarajan Amirthalingam Thandavarayan, Keith A. Youker, Xuehong Song, Di Ren, Ji Li, Raj Kishore, Prasanna Krishnamurthy, Lianchun Wang

**Affiliations:** ^1^Department of Molecular Pharmacology & Physiology, Morsani College of Medicine, Bryd Alzheimer's Research Institute, University of South Florida, Tampa, FL, United States; ^2^Center for Translational Medicine, Lewis Katz School of Medicine, Temple University, Philadelphia, PA, United States; ^3^Houston Methodist DeBakey Heart & Vascular Center, Houston, TX, United States; ^4^Department of Surgery, Morsani College of Medicine, University of South Florida, Tampa, FL, United States; ^5^Department of Biomedical Engineering, The University of Alabama at Birmingham, Birmingham, AL, United States

**Keywords:** STK35, diabetes, cardiac function, angiogenesis, serine threonine kinase, gene therapy

## Abstract

Diabetic cardiomyopathy (DCM) is characterized by microvascular pathology and interstitial fibrosis that leads to progressive heart failure. The mechanisms underlying DCM pathogenesis remain obscure, and no effective treatments for the disease have been available. In the present study, we observed that STK35, a novel kinase, is decreased in the diabetic human heart. High glucose treatment, mimicking hyperglycemia in diabetes, downregulated STK35 expression in mouse cardiac endothelial cells (MCEC). Knockdown of STK35 attenuated MCEC proliferation, migration, and tube formation, whereas STK35 overexpression restored the high glucose-suppressed MCEC migration and tube formation. Angiogenesis gene PCR array analysis revealed that HG downregulated the expression of several angiogenic genes, and this suppression was fully restored by STK35 overexpression. Intravenous injection of AAV9-STK35 viral particles successfully overexpressed STK35 in diabetic mouse hearts, leading to increased vascular density, suppression of fibrosis in the heart, and amelioration of left ventricular function. Altogether, our results suggest that hyperglycemia downregulates endothelial STK35 expression, leading to microvascular dysfunction in diabetic hearts, representing a novel mechanism underlying DCM pathogenesis. Our study also emerges STK35 is a novel gene therapeutic target for preventing and treating DCM.

## Introduction

Diabetes mellitus is a metabolic disease characterized by high blood glucose levels (1–3). Untreated high blood sugar in diabetes damages organs and tissues throughout the patient‘s body leading to complications such as cardiovascular disease. Heart disease, often presenting as cardiomyopathy, is the leading cause of death among patients with diabetes mellitus (4–6). Despite the recent advances in understanding diabetic cardiomyopathy (DCM), the full spectrum of contributing mechanisms and their relative contribution to DCM remains obscure. Also, no approved effective treatments for diabetes-induced cardiac dysfunction exists. Therefore, identifying novel mechanisms underlying DCM development and specific therapies targeting diabetes-induced cardiac dysfunction and subsequent heart failure are urgently needed (7).

The article "STK35 Gene Therapy Attenuates Endothelial Dysfunction and Improves Cardiac Function in Diabetes" was retracted in 2023. Reasons: duplicated images; unreliable data; unreliable results or conclusions.

The serine-threonine kinase 35 (STK35), also known as CLIK1 and STK35L1, is a novel kinase, mainly localizes in the nucleus and nucleolus and binds to nuclear actin (8–11). STK35 is a component of chromatin remodeling complexes (12) and, therefore, might directly influence the core transcription machinery and gene expression (13, 14). STK35 regulates multiple cellular functions such as cell migration, proliferation, survival, and angiogenesis (8, 15, 16). Moreover, the levels of STK35 were elevated in human colorectal cancer tissues (17) and altered in a rodent model of Parkinson's disease (18).

In the present study, we observed that the expression of STK35 is decreased in the diabetic human heart. High glucose (HG) decreased STK35 expression in mouse cardiac endothelial cells (MCEC) and MCEC proliferation, migration, and tube formation. Interestingly, replenishing STK35 expression restored HG-suppressed MCEC migration and tube formation. PCR array analyses revealed that HG-downregulated angiogenic gene expression was fully restored by STK35 overexpression. Furthermore, intravenous injection of AAV9-STK35 viral particles successfully overexpressed STK35 in the diabetic mouse heart and led to an increase in heart microvascular density, suppression of interstitial fibrosis, and amelioration of left ventricular functions. Altogether, our data reveal that HG-suppression of endothelial STK35 expression and associated microvascular dysfunction represents a novel mechanism underlying DCM pathogenesis.

## Materials and Methods

### Human Heart Tissues and Mouse Cardiac Endothelial Cells (MCEC)

Human heart tissue specimens were obtained from diabetic patients at the time of transplantation at the Houston Methodist DeBakey Heart and Vascular Center, Houston Methodist Hospital, Houston, Texas, and immediately frozen in liquid nitrogen and stored at −80°C until use. Non-diabetic hearts were obtained from donor hearts (not used for transplantation) and were collected and stored in the same manner. All tissues were collected under an approved protocol by the Houston Methodist Research Institutional Review Board. MCEC was purchased from Cedarlane (Cat#CLU510) and cultured in Dulbecco's modified Eagle's medium (DMEM, Invitrogen) with 10% fetal calf serum (ATCC) at 37°C and 5% CO_2_/95% air in a humidified environment.

The article "STK35 Gene Therapy Attenuates Endothelial Dysfunction and Improves Cardiac Function in Diabetes" was retracted in 2023. Reasons: duplicated images; unreliable data; unreliable results or conclusions.

### Streptozotocin-Induced Diabetic Mouse Model

Six-week-old male FVB/N mice were purchased from the Jackson laboratory. Animal studies were performed following relevant guidelines and regulations approved by the University of South Florida under ARRIVE guidelines. Animals were housed at constant RT (20 ± 1 °C) under a controlled 12-h light to 12-h dark cycle and had free access to water and a standard diet. The mice received a single *i.p*. injection of streptozotocin (100 mg/kg body weight, in 0.1 mol/l citric acid buffer, pH 4.5; Sigma–Aldrich, St Louis, MO, U.S.A.) to induce diabetes, or citric acid buffer vehicle (non-diabetic mice) (19–21). Diabetes was confirmed by measuring blood glucose from the saphenous vein using a glucometer (Roche, Basel, Switzerland). Mice with Streptozotocin-induced blood glucose levels >300 mg/dl were included in the diabetic groups.

### Adeno-Associated Virus Generation and Administration

The customized STK35-GFP-CMV-AAV Vector (mouse CMV) construct was purchased from ABM company (catalog numberAAV0047594) and cloned into a recombinant adeno-associated virus (rAAV) plasmid with a GFP, packaged into pseudotype-9 capsids (rAAV9) (Supplementary Figure 1) (22, 23). Briefly, The STK35-GFP-CMV-AAV Vector was generated by transfection of the STK35 isoform a-eGFP plasmid with the helper plasmids pXX6, pAAV9, and PEI solution in 20 15 cm plates of human embryonic kidney-derived 293 cells (HEK 293) at 75% confluency. After 72 h, the transfected HEK 293 cells were harvested and pelleted by centrifugation. After resuspension in lysis buffer with protease inhibitors, the HEK 293 cells were lysed via three freeze/thaw cycles in dry ice and 100% ethanol bath. The constructed viral vector was purified by pipetting lysis solution above a four iodixanol gradient in 39 mL Quick-Seal^®^ Beckman tubes. The tubes were centrifuged in type 70 Ti Beckman rotor at 60,000 rpm for 2 h. The iodixanol gradient layer containing the viral vector was extracted and purified by 5 PBS washes in Apollo concentrators. A dot-blot assay was performed to determine the final concentration of the viral vector using the known STK35 plasmid concentrations as the standards with a denatured probe. rAAV9-STK35 (2 × 10^11^ virus in 150 μl of saline), transgene-null vector (rAAV9-null), or saline vehicle control were administered via a single tail-vein injection (24).

The article "STK35 Gene Therapy Attenuates Endothelial Dysfunction and Improves Cardiac Function in Diabetes" was retracted in 2023. Reasons: duplicated images; unreliable data; unreliable results or conclusions.

### High Glucose Treatment in MCEC

To mimic hyperglycemia, MCEC at confluent density were cultured for 48 h in DMEM media supplemented with 30 mmol/L D-glucose (HG; high glucose). D-Mannitol was used as an osmotic control (NG; normal glucose).

### RNA Isolation and Quantitative Reverse Transcription PCR (qRT-PCR)

Briefly, cells or tissues were homogenized using a trizol lysis reagent. RNA was isolated from the homogenized samples using the miRNeasy Mini Kit (Qiagen). First-strand cDNA was synthesized using the TaqMan miRNA Reverse Transcription Kit following the vendor's instructions (Applied Biosystems, Foster City, CA). qRT-PCR was performed using the Step-One Plus system (Life Technologies) following the manufacturer's instructions. The expression of the target gene was normalized to the GAPDH for comparison (25–27).

### Western Blot Analysis

Western blotting of protein lysate from cultured cells was performed as previously described (27–29). Briefly, cells were homogenized in lysis buffer (Cell Signaling Technology, MA, USA) containing 20 mmol/l Tris-HCl [pH 7.5], 150 mmol/l NaCl, 2.5 mmol/l sodium pyrophosphate, 1 mmol/l β-glycerophosphate, 1 mmol/l sodium orthovanadate, 1 μg/ml leupeptin, 1 mmol/l ethylenediaminetetraacetic acid, 1 mmol/l ethylene glycol tetraacetic acid, 1% Triton X-100 and protease inhibitors. Equal amounts of protein were separated by 10% SDS-PAGE and blotted onto polyvinylidene difluoride membranes (Bio-Rad, Hercules, CA). The blots were incubated with antibodies against STK35 (Cat#ab37974; Abcam, USA) and developed with an enhanced chemiluminescence detection system (Amersham, Piscataway, NJ).

### Knockdown and Overexpression of STK35 in MCEC

To knockdown *STK35* in MCEC, the cells were transduced with lentiviral-based *STK35* specific short hairpin RNA (mission shrna transduction particles NM_183262/TRCN0000026703) (*STK35*-shRNA; Sigma Aldrich, MO) or non-specific control-shRNA (SHC005V) (5 MOI, multiplicity of infection) in the presence of hexadimethrine bromide (6 μg/ml; increases transduction efficiency) as described in our previous publication (28). *STK35* was overexpressed in MCEC by transfecting the cells with pcDNA3.4-TOPO-STK35 from Thermo-Fisher. Transfection efficiency was determined by measuring STK35 expression by qRT-PCR and Western blot analyses.

### Cell Proliferation

The mitogenic activity of STK35 on MCEC was measured by the Cell Counting Kit 8 (WST-8 / CCK8) (ab228554; Abcam, USA). In brief, the STK35 knockdown or STK35 overexpression MCECs at 10^3^ per well were seeded into a 96-well plate and cultured for 48 h. After the addition of the CCK8 solution and incubation for an additional 1-h, Absorbance at 450 nm wavelength was measured in a plate reader (Bio-Tek). The cell proliferation rate was determined by A450nm minus the background control signal.

The article "STK35 Gene Therapy Attenuates Endothelial Dysfunction and Improves Cardiac Function in Diabetes" was retracted in 2023. Reasons: duplicated images; unreliable data; unreliable results or conclusions.

### Cell Trans-Well Migration

The migration of MCEC toward VEGF165 stimulation was performed in a 24-well Boyden chamber Transwell plate (27). Briefly, 20 ng/ml VEGF165 in 600 μl of chemotaxis buffer (serum-free DMEM, 0.1% BSA) was added to the lower compartment. MCEC (1 × 10^5^ cells) in 100 μl of chemotaxis buffer were added to the upper compartment (transwell inserts with 8-μm pores [Costar]). After incubation at 37°C for 18 h, the filters were removed. The cells that migrated through the pores to the bottom chamber were stained with Hema-3^®^ stain kit (Millipore, Billerica, MA) counted manually in 5 random fields in each well. All groups were studied at least in triplicate.

### MCEC Tube Formation

MCEC expressing STK35-shRNA, pcDNA3.4-TOPO-STK35, or respective scramble control were cultured for 48 h. Then, the conditioned media was collected and mixed in equal quantities of fresh medium (1:1), and 300 ul of the medium with 1.5 × 10^4^ MCEC per well was seeded in a 48-well plate precoated with 40 ul per well growth factor reduced Matrigel (BD Falcon). After 6 h in culture, capillary-like tube formation was photographed by a phase-contrast microscope. The cumulative length of the formed tubes was quantified using ImageJ software.

### Angiogenesis PCR Array

To determine the potential molecules by which STK35 promotes angiogenesis, MCEC with STK35 overexpression were cultured in normal or high glucose for 48 h, and then collected for expression profiling of genes that modulate angiogenesis using Mouse Angiogenesis RT^2^ Profiler™ PCR Array (Qiagen, PAMM-024Z) according to the manufacturer's instruction.

### Echocardiography

Transthoracic two-dimensional M-mode echocardiogram was obtained using Vevo 770 (VisualSonics, Toronto, Canada) equipped with a 30 MHz transducer. Echocardiographic studies were performed before (baseline) and at 8 weeks post-rAAV9-STK35 *i.v*. injection. The mice were anesthetized with a mixture of 1.5% isoflurane and oxygen (1 l/min). M-mode tracings were used to measure the end-systolic diameter (LVESD), and end-diastolic diameter (LVEDD) and percent ejection fraction (%EF) was calculated as previously described (27, 28).

### Cardiac Fibrosis Assessment

Histopathological assessment of cardiac fibrosis was performed as previously described (27, 28). The hearts were fixed with 10% buffered formalin and paraffin-embedded. The cardiac fibrosis area was quantified on Masson's trichrome-stained sections by using NIH's ImageJ software.

### Immunofluorescence Staining of Tissue Sections

Immunofluorescence staining of tissue sections was performed as described previously (27, 28). Tissue sections were permeabilized and counter-stained with 4′, 6-diamidino-2-phenylindole (DAPI, 1:5000, Sigma Aldrich, St Louis, MO), and sections were examined with a fluorescent microscope (Nikon ECLIPSE TE200, Japan). The number of CD31^+^ stained capillaries was assessed in 10 randomly selected high-power visual fields.

The article "STK35 Gene Therapy Attenuates Endothelial Dysfunction and Improves Cardiac Function in Diabetes" was retracted in 2023. Reasons: duplicated images; unreliable data; unreliable results or conclusions.

### Statistical Analysis

Data are presented as mean ± SE. Between two groups of mice, an unpaired Student's *t*-test was performed to determine statistical significance. When involving more than two groups, ANOVA with Tukey *post-hoc* test was used to analyze the data. Probability (P) values of <0.05 were considered a significant difference.

## Results

### STK35 Expression Decreases in the Diabetic Human Heart

In previous studies, we uncovered STK35 plays a key role in maintaining the functions of human CD34+ progenitor cells in the ischemia heart (27). To explore if STK35 is dysregulated in diabetes and contributes to DCM, we initially analyzed publicly available mRNA expression data from 7 human diabetic hearts and 5 human non-diabetic heart controls (GSE26887). We found a significant decrease in STK35 mRNA expression in human diabetic hearts compared to human non-diabetic hearts (Figure 1A). To confirm this finding, we analyzed 5 diabetic and 4 non-diabetic human cardiac biopsies that were collected at the Houston Methodist DeBakey Heart & Vascular Center. The patient information is detailed in Supplementary Table 1. In immunostaining, we observed a decrease in the number and intensity of STK35 positive cells in the diabetic heart as compared to the control non-diabetic human heart (Figure 1B). Similarly, western blotting and qRT-PCR analyses detected a marked reduction of STK35 at protein and mRNA levels, respectively, in the diabetic human heart compared to non-diabetic human heart tissue (Figures 1C,D). These findings conclude that STK35 expression is decreased in the human diabetic heart.

**Figure 1:** STK35 expression is decreased in the diabetic human heart. **(A)** STK35 expression in diabetic human heart from publicly available RNA sequence data. STK35 expression in the GSE26887 datasheet includes 5 non-diabetic human hearts and 7 diabetic human heart tissues. **(B)** Immunohistochemistry staining showed a decrease in STK35 expression in the diabetic human heart compared to the non-diabetic human heart. Scale bar: 100 μm. **(C)** Western blotting and quantification analyses of STK35 expression in both non-diabetic and diabetic human hearts. **(D)** qRT-PCR data showing a decrease in STK35 mRNA expression in the diabetic human heart compared to the non-diabetic human heart. Data were normalized against GAPDH mRNA. *n* = 4, non-diabetic human heart; *n* = 5, diabetic human heart. **P < 0.01, and ***P < 0.001.

The article "STK35 Gene Therapy Attenuates Endothelial Dysfunction and Improves Cardiac Function in Diabetes" was retracted in 2023. Reasons: duplicated images; unreliable data; unreliable results or conclusions.

### Diabetic Condition Decreases STK35 Expression in Mouse Cardiac Endothelial Cells

Our clinical patient specimen studies determined that STK35 expression is decreased in the human diabetic hearts, but it remains unknown the cell types that showed the most significant STK35 expression reduction in DCM and if the expression downregulation is induced by hyperglycemia (a diabetic condition). In the initial study, we mined cell-type STK35 expression in the human heart in THE HUMAN PROTEIN ATLAS (https://www.proteinatlas.org/ENSG00000125834-STK35/celltype). We found STK35 expression is the highest in the cardiac endothelial cells and fibroblasts (Figure 2A). Adult mouse heart shows a similar cell-type STK35 mRNA expression pattern (30) (data not shown) (https://tabula-muris.ds.czbiohub.org/). Cardiac endothelial cells are more abundant than fibroblasts in human and mouse hearts, and our previous study showed that STK35 promotes human umbilical endothelial cells (HUVEC) proliferation and tube formation (27). Therefore, we focused our study on STK35 expressed in cardiac endothelial cells and further tested if hyperglycemia downregulates STK35 expression in MCEC. We treated MCEC with HG (30 mM/L glucose for 48 h), a condition that mimics hyperglycemia. Immunofluorescence staining observed a decrease of STK35 in the HG-treated MCEC compared to normal glucose (NG)-treated MCEC (Figure 2B). Similarly, RT-PCR and western blot analyses determined a significant decrease in STK35 expression in HG-treated MCEC cells at mRNA and protein levels, respectively (Figures 2C,D). These data, together, demonstrate that hyperglycemia directly downregulates STK35 expression in MCEC under diabetic conditions.

**Figure 2:** High glucose downregulates STK35 expression in mouse cardiac endothelial cells. **(A)** Cell type-specific STK35 mRNA expression in the adult human heart. The STK35 mRNA levels in different human heart cell types were determined by mining single-cell RNAseq data deposited in THE HUMAN PROTEIN ATLAS database (https://www.proteinatlas.org/ENSG00000125834-STK35/celltype/heart+muscle). The different heart cell types are colored according to clusters and are represented using Uniform manifold approximation and projection (UMPA). The cell-type expressions of STK35 mRNA were represented by the mean protein-coding transcripts per million (pTPM). **(B)** Immunofluorescence staining observed decreased STK35 expression in high glucose treated MCEC compared to MCEC treated with normal glucose. Scale bars: 50 μm. **(C)** Western blotting analysis of STK35 expression in MCEC treated with high glucose. **(D)** qRT-PCR data showing decreased *STK35* mRNA expression in high glucose-treated MCEC compared to MCEC treated with normal glucose. Data were normalized to GAPDH mRNA. *n* = 3, *P < 0.05 and **P < 0.01.

The article "STK35 Gene Therapy Attenuates Endothelial Dysfunction and Improves Cardiac Function in Diabetes" was retracted in 2023. Reasons: duplicated images; unreliable data; unreliable results or conclusions.

### STK35 Knockdown Inhibits MCEC Proliferation, Migration, and Tube Formation

To evaluate the functional consequence of the downregulated STK35 expression in MCEC, we knocked down STK35 in MCEC using lentiviral-based shRNA against STK35. Western blot analysis indicated that the lentiviral STK35 shRNA successfully suppressed STK35 protein expression (Figure 3A), and this was further confirmed in qRT-PCR analysis (Figure 3B). In cell function analysis, the STK35-knockdown inhibited VEGF-induced MCEC proliferation and trans-well migration, compared to mock shRNA control (Figures 3C,D). Furthermore, we observed that the STK35-knockdown inhibited MCEC's ability to form vascular tubes in culture (Figure 3E). These data illustrate that the downregulation of STK35 disturbs MCEC functions.

**Figure 3:** STK35 knockdown impairs MCEC proliferation, migration, and tube formation. **(A)** Western blotting and **(B)** qRT-PCR analyses showing STK35 was knocked down in MCEC transduced with lentiviral STK35 shRNA. Data were normalized to β-actin and GAPDH, respectively. *n* = 3. **(C)** MCEC proliferation (*n* = 8). **(D)** Boyden chamber migration assay determining the migratory responses of lentiviral STK35 shRNA or scrambled control shRNA transduced MCEC toward VEGF gradient (*n* = 6). **(E)** Matrigel tube formation assay. Tubes formed by MCEC transduced with lentiviral STK35 shRNA or scrambled control shRNA were imaged, and tube length was quantified. *n* = 6. ****P < 0.0001.

### STK35 Overexpression Normalizes HG-Induced MCEC Dysfunction

To test if an increase of STK35 expression will reverse hyperglycemia-induced MCEC dysfunctions, we overexpressed STK35 in HG-treated MCEC by transfecting the cells with pcDNA3.4-TOPO-STK35. Western blot and qRT-PCR analyses showed the pcDNA3.4-TOPO-STK35 transfection restored STK35 protein and mRNA levels in the HG-treated MCEC (Figures 4A,B). In a modified Boyden chamber migration assay, the pcDNA3.4-TOPO-STK35-expression substantially restored HG-suppressed MCEC migration in response to VEGF stimulation (Figure 4C). The pcDNA3.4-TOPO-STK35 overexpression also restored MCEC tube formation that is inhibited by HG treatment (Figure 4D). These results showed that increasing STK35 expression restores HG-induced MCEC dysfunctions. To determine the effect STK35 on angiogenesis-related genes expression, we carried out mouse angiogenesis PCR array analysis (Supplementary Table 2 shows the gene list). HG treatment downregulated the expression of some notable angiogenic genes, including connective tissue growth factor (ctgf), VEGF-A, MMP9, and IL-6, and the downregulation of these angiogenic genes were restored and even increased by STK35 overexpression (Figure 5A). We analyzed the mRNA expression of the angiogenic genes in publicly available mRNA expression data from 7 human diabetic hearts and 5 human non-diabetic hearts (GSE26887). We observed similar decreases of the angiogenic gene mRNA expression in human diabetic hearts compared to non-diabetic human hearts (GSE26887) (Figure 5B). These results show that STK35 overexpression restores the angiogenic gene expressions suppressed by hyperglycemia, thus ameliorating MCEC dysfunction in high glucose conditions.

The article "STK35 Gene Therapy Attenuates Endothelial Dysfunction and Improves Cardiac Function in Diabetes" was retracted in 2023. Reasons: duplicated images; unreliable data; unreliable results or conclusions.

**Figure 4:** STK35 overexpression restores high glucose-induced impairment of MCEC migration and vascular tube formation. **(A,B)** Western blotting and qRT-PCR analyses showing transfection with pcDNA3.4-TOPO-STK35 over-expressed STK35 in MCEC. Data normalized to β-actin and GAPDH, respectively. *n* = 3. **(C)** Boyden chamber migration assay determining the migratory responses of STK35 shRNA or scrambled control shRNA transduced MCEC toward VEGF gradient in high glucose culture condition. **(D)** Matrigel tube formation assay. Tubes formed by MCEC transfected with pcDNA3.4-TOPO-STK35 or scramble control plasmid in high glucose culture were imaged, and tube length was quantified. *n* = 6. *P < 0.05, **P < 0.01, ***P < 0.001, and ****P < 0.001.

**Figure 5:** Overexpression of STK35 restores high glucose-induced downregulation of pro-angiogenic gene expression. **(A)** Mouse PCR angiogenesis array showing high glucose downregulates several angiogenic factor expressions in MCEC, including *Ctgf* and *Vegfa*, whereas the downregulations were restored by STK35 overexpression. The gene expression data were normalized to normal glucose control and are presented as fold change. **(B)** Angiogenic gene expression in diabetic human hearts from publicly available RNA sequence data (GSE26887).

### AAV9-STK35 Protects Against Diabetes-Induced Cardiac Dysfunction and Left Ventricle Remodeling

DCM is characterized by microvascular pathology and interstitial fibrosis, which lead to progressive heart failure. To determine if restoration of STK35 expression in MCEC will ameliorate DCM, diabetic mice were injected *i.v*. with AAV9-STK35. Eight weeks later, the mice were examined. AAV9-STK35 injection led to abundant STK35 expression in the heart, mainly in the vasculature, as determined by immunofluorescence staining (Figure 6A). CD31 immunostaining and Trichrome-staining showed that AAV9-STK35 administration significantly increased cardiac vascular density, whereas decreased cardiac fibrosis in the diabetic hearts (Figures 6B,C). Echocardiography analyses show that AVV9-STK35 overexpression increased both percent left ventricular ejection fraction and percent fractional shortening of the diabetic mouse group (Figure 6D). Together, these data suggest that overexpression of STK35 increases myocardial vascularization and blocks myocardial fibrosis, thus leading to amelioration of left ventricular function in diabetic mice.

The article "STK35 Gene Therapy Attenuates Endothelial Dysfunction and Improves Cardiac Function in Diabetes" was retracted in 2023. Reasons: duplicated images; unreliable data; unreliable results or conclusions.

**Figure 6:** AAV9-mediated overexpression of STK35 enhances neovascularization, reduces fibrosis, and improves left ventricular function in diabetic mice. **(A)** Immunohistochemistry staining shows AAV-9-STK35 expression in diabetic mouse hearts. STK35. **(B)** Representative images of the capillary vasculature in diabetic mouse heart treated with saline or i*.v*. injected with scramble AAV9 or AAV9-STK35. Capillary vessels were stained with CD31+ (red), and nuclei were counterstained with DAPI (blue). Graph depicting capillary density as the percentage of CD31+ cells. **(C)** Trichrome staining and percentage of fibrosis in the diabetic heart from the mice treated with saline or i*.v*. injected with scramble AAV9 or AAV9-STK35. Scale bar 100 μm. **(D)** Quantitative analyses of percent ejection fraction (%EF) and percent fractional shortening (%FS). (*n* = 4); *P < 0.05 and **P < 0.01.

## Discussion

Despite receiving significant research attention over several decades, DCM remains the leading cause of death among diabetic patients (31). Further studies to understand the full spectrum of potential contributing mechanisms and the development of therapies that target diabetes-induced cardiac dysfunction and subsequent heart failure are urgently needed. In the present study, we uncovered STK35, a novel kinase that is most abundantly expressed in heart endothelial cells, is downregulated in DCM. Our *in vitro* studies established hyperglycemia downregulates STK35 in MCEC and disturbs MCEC functions. Mechanistically, hyperglycemia downregulates STK35 leading to suppression of the expression of several potent angiogenic genes. More importantly, cardiac-targeted expression of STK35 exerts a marked beneficial action, including increasing cardiac vascular density, attenuating cardiac remodeling, and ameliorating cardiac function in a mouse model of diabetes mellitus. This mouse model study highlights STK35 as a novel gene therapy target for preventing and treating human DCM.

Serine/threonine kinases (STKs) play critical pathophysiological roles through the phosphorylation and activation of relevant effectors, such as cell-cycle regulators, growth factors, and transcription activators, to regulate signaling pathways and cellular homeostasis (17, 32). Currently, the detailed biological functions of STK35 are still being investigated. STK35 has been shown to regulate the cell cycle, and its abnormal cellular levels are implicated in various human diseases, including cancer and Parkinson's disease (9, 11). In the current study, we uncovered that STK35 levels are decreased in DCM in patients. In a normal human heart, STK35 expression is most abundant in endothelial cells and fibroblasts and low level of expression in cardiomyocytes. In the current study, we have not further investigated cell type-specific expression of STK35. This information might be critical to better understand the functions of STK35 in heart hemostasis and DCM pathogenesis. We will address this issue in our future study. Early studies observed STK35 regulates the human umbilical vein endothelial cell cycle and promotes migration (9). Our previous studies observed STK35 enhances human CD34+ endothelial progenitor cell angiogenic activity and neovascularization of heart after ischemia-reperfusion injury in a mouse model (27). Our present study demonstrated that STK35 promotes angiogenesis of MCEC and neovascularization in diabetic mouse hearts, directly showing that STK35 possesses a proangiogenic function.

The article "STK35 Gene Therapy Attenuates Endothelial Dysfunction and Improves Cardiac Function in Diabetes" was retracted in 2023. Reasons: duplicated images; unreliable data; unreliable results or conclusions.

Multiple clinical and experimental studies have established the comprised cardiac structure and function are independent of the macrovascular complications of diabetes, including hypertension, coronary artery disease, and atherosclerosis (33–37), but are associated with microvascular pathology (38). Restoration of microvascular homeostasis recovers cardiac function in DCM (38, 39). Evaluation of the pathogenesis of DCM in a streptozotocin-induced diabetic rat model demonstrates that downregulation of myocardial VEGF expression preceded all other features of DCM and followed the order of increased apoptosis of endothelial cells, decreased numbers of circulating endothelial progenitor cells, decreased capillary density, and impaired myocardial perfusion along with apoptosis and necrosis of cardiomyocytes, fibrosis and progressive heart dysfunction (38). Replenishing myocardial VEGF expression increased capillary density, decreased apoptosis of endothelial cells and cardiomyocytes, attenuated *in situ* differentiation of bone marrow-derived endothelial progenitor cells into endothelial cells, and significant improvements in cardiac function, thus suggesting the critical role of VEGF in the pathophysiology of DCM (38). This rat model study suggested that progressive attenuation of myocardial VEGF expression is central for DCM pathogenesis. However, how myocardial VEGF expression is attenuated in DCM remains unknown. In the present study, we observed decreased STK35 expression in DCM, HG downregulates STK35 and VEGF expression in MCEC, and the HG-suppressed VEGF expression was restored by STK35 overexpression. This data suggests the functional consequence of the detrimental effect of hyperglycemia in diabetes: HG downregulates STK35 in MCEC, leading to suppression of VEGF expression and the ensuing cardiac vascular pathology in DCM. Considering the central role of VEGF expression in DCM, we postulate that decreased STK35 expression in DCM is the major upstream signaling that leads to suppressed VEGF signaling in the disease. Our study also observed that overexpression of STK35 restored the expression of other angiogenic genes, including ctgf, MMP9, and IL-6, which may contribute to the normalization of hyperglycemia-induced cardiac endothelial cell dysfunction and maintains hemostasis of cardiac vasculature. Our data highlights that alterations of myocardial STK35 expression are a seminal event of vascular dysfunction in DCM.

The article "STK35 Gene Therapy Attenuates Endothelial Dysfunction and Improves Cardiac Function in Diabetes" was retracted in 2023. Reasons: duplicated images; unreliable data; unreliable results or conclusions.

There has been a lack of effective treatments for diabetes-induced cardiac dysfunction. The treatment of diabetes by controlling blood glucose has failed to improve cardiac function or reduce the risk of heart failure (40–42). The conventional therapy for heart failure is the same, whether or not the patient has diabetes. Overexpression of VEGF and decorin, a type of small leucine-rich proteoglycan, in the heart promoted angiogenesis and ameliorated DCM-associated cardiac pathology in mouse models (38, 39). In the present study, we used rAAV9-STK35 and found increased expression of STK35 in the heart, which increased microvascular density, suppressed fibrosis, and ameliorated heart functions in diabetic mice, suggesting that STK35 is a novel gene target for preventing and treating DCM.

## Conclusion

Our findings suggest that hyperglycemia downregulates STK35 expression in the heart, leading to suppression of angiogenic gene expression, disruption of microvascular homeostasis in the myocardium, and the subsequent left ventricle dysfunction in DCM. Our findings also emerge targeting STK35 may be effective in preventing and treating human DCM.

## Data Availability Statement

The original contributions presented in the study are included in the article/Supplementary Material, further inquiries can be directed to the corresponding author/s.

## Ethics Statement

The studies involving human participants were reviewed and approved by Houston Methodist DeBakey Heart and Vascular Center, Houston Methodist Hospital, Houston, Texas. The patients/participants provided their written informed consent to participate in this study. The animal study was reviewed and approved by University of South Florida under ARRIVE guidelines. Written informed consent was obtained from the individual(s) for the publication of any potentially identifiable images or data included in this article.

The article "STK35 Gene Therapy Attenuates Endothelial Dysfunction and Improves Cardiac Function in Diabetes" was retracted in 2023. Reasons: duplicated images; unreliable data; unreliable results or conclusions.

## Author Contributions

DJ, YZ, MW, KN, MC, RT, KY, XS, DR, JL, RK, and LW conducted the experiments, acquisition, and analysis of the results. DJ, PK, and LW designed the experiments, interpreted the data, and drafted the manuscript. All authors reviewed the results and approved the final version of the manuscript.

## Funding

This work was supported by NIH R01 HL093339, U01 CA225784, 1RF1 AG074289 and 1RF1 AG069039 (LW), American Heart Association postdoctoral grant 16POST30780010 (DJ) and R01GM124108 and R01HL158515 (JL).

## Conflict of Interest

The authors declare that the research was conducted in the absence of any commercial or financial relationships that could be construed as a potential conflict of interest.

## Publisher's Note

All claims expressed in this article are solely those of the authors and do not necessarily represent those of their affiliated organizations, or those of the publisher, the editors and the reviewers. Any product that may be evaluated in this article, or claim that may be made by its manufacturer, is not guaranteed or endorsed by the publisher.

## Abbreviations

DCM: diabetic cardiomyopathy
HG: high glucose
MCEC: mouse cardiac endothelial cells
NG: normal glucos
VEGF: vascular endothelial growth factor
CTGF: connective tissue growth factor.
